# microRNA-155 Modulates Hepatic Stellate Cell Proliferation, Apoptosis, and Cell Cycle Progression in Rats With Alcoholic Hepatitis *via* the MAPK Signaling Pathway Through Targeting SOCS1

**DOI:** 10.3389/fphar.2020.00270

**Published:** 2020-04-07

**Authors:** Dengtao Liu, Ping Han, Chunhai Gao, Wei Gao, Xiaocui Yao, Shulan Liu

**Affiliations:** ^1^ Clinical Laboratory, Linyi People’s Hospital, Linyi, China; ^2^ Department of Pulmonary and Critical Care Medicine, Linyi People’s Hospital, Linyi, China; ^3^ Department of Imaging, Linyi People’s Hospital, Linyi, China

**Keywords:** microRNA-155, suppressor of cytokine signaling 1, mitogen-activated protein kinase signaling pathway, alcoholic hepatitis, hepatic stellate cell, proliferation and apoptosis

## Abstract

The aim of this study was to investigate the regulatory function of the non-coding microRNA-155 (miR-155) and suppressor of cytokine signaling 1 (SOCS1) in alcoholic hepatitis (AH) and its potential mechanism associated with the mitogen-activated protein kinase (MAPK) signaling pathway. Levels of alanine aminotransferase (ALT), aspartate aminotransferase (AST), albumin (ALB), total bilirubin (TBIL), malondialdehyde (MDA), and superoxide dismutase (SOD) were measured in a rat model of AH. The biological prediction website microRNA.org and dual-luciferase reporter gene assay were used to identify whether SOCS1 was a direct target of miR-155, and the effects of miR-155 and SOCS1 on the viability, cycle progression, and apoptosis of hepatic stellate cells were assessed using RT-qPCR, Western blot assay, MTT assay, Annexin V/PI double staining, and PI single staining. The levels of ALT, AST, MDA, and TBIL and the liver cell morphology were all prominently changed in AH model rats. miR-155 suppressed SOCS1 by specifically binding to SOCS1-3’-UTR to activate the MAPK signaling pathway. SOCS1 had low expression while miR-155 was highly expressed in AH rats. miR-155 promoted hepatic stellate cell viability and cycle progression and reduced cell apoptosis by silencing SOCS1. Together, we find that silenced miR-155 could upregulate SOCS1 and inactivate the MAPK signaling pathway, thereby inhibiting the proliferation of alcoholic hepatic stellate cells and promoting cell apoptosis.

## Introduction

Liver cancer is the sixth most frequently diagnosed cancer and ranks fourth worldwide as a cause of mortality (Bray et al., 2018). Alcoholic liver disease (ALD) can bring the morbidities of fibrosis and cirrhosis and is one of the major causes of chronic liver cancer (Gao and Bataller, 2011). The spectrum of ALD mainly encompasses alcoholic hepatitis (AH), alcoholic fatty liver disease (AFLD), and chronic ALD. AH, as a uniquely alcohol-associated liver disease, causes acute liver inflammation as a result of prolonged and heavy alcohol abuse (Im, 2019). Moreover, AH is characterized by steatosis, fibrosis, necroinflammation, and potential complications to liver disease (Pavlov et al., 2017). In the past, study of the pathogenesis of AH chiefly focused on factors such as ethanol metabolism, malnutrition, abnormal methionine metabolism, and production of endotoxins. Moreover, the treatment of AH primarily includes symptomatic treatment with corticosteroids, pentoxifylline, nutritional support, and abstinence counseling (Gao and Bataller, 2011).

As critical regulators of cellular proliferation and differentiation, non-coding microRNAs (miRNAs or miRs) have great potential in the modulation of disease pathogenesis and can be regarded as biomarkers or therapeutic targets. For instance, miR-182 expression was demonstrated to be correlated with the degree of disease severity and liver disease injury and proved to be a biomarker and therapeutic target for AH (Blaya et al., 2016). Another research study has demonstrated that silencing miR-21 in hepatic stellate cells may prevent the progress of ALD-like histopathology (Wu et al., 2018). miR-155 is a regulator of inflammation in alcohol-related liver injuries and is highly expressed in liver disease (Bala et al., 2012), thus serving as a key miRNA in ALD development (Hartmann and Tacke, 2016). In addition, miR-155 was verified to be an alcohol-related mediator in ALD progression (Babuta et al., 2019). Based on these research results, we predicted that miR-155 was involved in AH.

Suppressor of cytokine signaling-1 (SOCS1), also known as JAK-binding protein, is an intracellular protein involved in inflammatory responses. The mRNA expression level of SOCS1 in chronic hepatitis C is closely correlated with the occurrence of cirrhosis (Pascarella et al., 2013). Another study indicated that SOCS1 was associated with the development of non-alcoholic fatty liver disease (Younossi et al., 2009). Moreover, by directly targeting SOCS1, miR-155 may serve as a pro-proliferative modulator with the ability to promote liver regeneration (Lin et al., 2018). These research findings contributed to the formulation of our hypothesis that miR-155 might target SOCS1 to participate in the regulation of AH. Other results document that SOCS1 can inactivate the mitogen-activated protein kinase (MAPK) signaling pathway to exert anti-proliferative effects on gastric cancer cells (Souma et al., 2012). The MAPK signaling pathway, especially upon activation by lipopolysaccharide (LPS), plays an active role in liver inflammation and injury (Mandrekar and Szabo, 2009; Liu H. et al., 2015). However, it is still enigmatic whether miR-155 participates in AH development by regulating the MAPK signaling pathway *via* SOCS1. In this regard, the current study aims to investigate the regulatory function of miR-155 and SOCS1 in hepatic stellate cells and in AH model rats and to probe the potential disease mechanism associated with the MAPK signaling pathway. In this study, we measured changes in the expression of miR-155, SOCS1, and MAPK signaling pathway-related genes in liver tissues of AH model rats. We then altered SOCS1 and miR-155 expression in hepatic stellate cells isolated from AH rats to investigate their impacts on the MAPK signaling pathway and the biological properties of the cells.

## Materials and Methods

### Ethics Statement

Animal experiment protocols were approved by the Experimental Animal Ethics Committee of Linyi People’s Hospital. All animal experiments were performed in accordance with the Guide for the Care and Use of Laboratory Animals published by the National Institutes of Health (NIH Publications No. 8023, revised 1978) and in accordance with local principles of the management and use of laboratory animals. Appropriate measures were taken to minimize the numbers of animals used as well as their suffering.

### Development of Rat Models With AH

Twenty Sprague-Dawley (SD) rats (ten males, ten females) (weighing 190 to 210 g, aged 6 to 7 weeks) were randomly assigned to normal (n = 8) and AH model groups (n = 12). They were housed in a specific pathogen-free (SPF) animal laboratory environment at 22–25°C and a relative humidity of 60-65%. Rats were fed ad libitum during seven days of acclimation, whereupon the AH rats began additional gavage with 9 mL/kg/day white wine according to their body weight for modeling at intervals of 8 hours for 6 weeks.

The physiological status and tissue structure of rats were observed to judge whether the modeling was successful according to the following criteria: (1) physiological status: asymptomatic performance or right upper abdominal distension, irritability, loss of appetite, weight loss, listlessness, and other symptoms; (2) physiological and biochemical indexes: the plasma levels of alanine aminotransferase (ALT), aspartate aminotransferase (AST), albumin (ALB), total bilirubin (TBIL), malondialdehyde (MDA), and superoxide dismutase (SOD) were measured. Animals with increased levels of ALT, AST, MDA, and TBIL, decreased levels of SOD and ALB, and AST/ALT > 2, were judged to be successful (Liu S. et al., 2015); (3) pathological examination: after hematoxylin and eosin (HE) staining, the structure of liver tissue slices was observed under a light microscope to confirm the model (O’Brien et al., 2011). Eight rats with AH were randomly selected for subsequent experiments.

### Specimen Collection and Preparation

After the last gavage treatment, the rats fasted for 12 hours. Under anesthesia by intraperitoneal pentobarbital injection (0.3 mL/100 g body weight), blood was drawn from the abdominal aorta and transferred to disposable centrifuge tubes, whereupon the rats were euthanized. After standing at room temperature, the blood was centrifuged at 3000 rpm for 20 min, and the serum was separated and refrigerated at -20°C. The livers were dissected and repeatedly washed in physiological saline until there was no evident congestion. After surface drying with filter paper, livers were weighed, and a portion (1.0 × 1.0 × 0.5 cm) was dissected and fixed by immersion in 10% formaldehyde.

### Detection of Physiological and Biochemical Indexes

The contents of ALT, AST, ALB, TP, ADH, and TBIL were detected using an RA1000 automatic biochemical analyzer (Olympus, Tokyo, Japan). The levels of MDA and SOD were measured by means of an assay kit (Solarbio Science & Technology Co., Ltd., Beijing, China).

### Hematoxylin and Eosin (HE) Staining

The formaldehyde-fixed liver specimen was conventionally dehydrated in an ascending concentration series of ethanol (70, 80, 90, 95, and 100%; one hour per bath), cleared twice in dimethylbenzene (30 min each), embedded in paraffin, and sliced to a thickness of 4mm. After being baked at 60°C for an hour, the slices were dewaxed with xylene and rehydrated with the reversed ethanol gradient. The slices were then stained with hematoxylin for ten minutes, differentiated with 1% hydrochloric acid in alcohol for 20 seconds, and reverted to blue color by immersion in 1% ammonium hydroxide for 30 seconds. The slices were stained with eosin for three minutes, dehydrated with gradient ethanol (two minutes each time), cleared twice with xylene (five minutes each time), mounted with neutral balsam, and observed and photographed at 40 × magnification under an ordinary optical microscope (Olympus Optical Co., Ltd, Tokyo, Japan).

### Culture and Identification of Rat Hepatic Stellate Cells

Rats with AH and normal rats were anesthetized with pentobarbital (5 mg/100 g body weight) by intraperitoneal injection. The rats were disinfected with 5% alcohol, and the abdomen in the right middle was opened to expose the liver. A pre-warmed ethylene glycol-bis (β-aminoethyl ether)-N, N, N’, N’-tetraacetic acid solution was instilled for ten minutes, followed by 0.5 mg/m LIV-type collagenase for 15 minutes. After the liver was removed and minced, 50 mL of 0.5 mg/mL collagen enzyme solution was added. The mixture was shaken and detached for 30 minutes at 37°C, and the suspension was collected after filtration through a 200-mesh polyethylene net. After centrifugation at 500 × g for seven minutes at 4°C, the supernatant was discarded, and the cell pellet was collected. This was resuspended in buffer in a 50 mL sterile centrifuge tube and recentrifuged for collection of the washed cell pellet. After being combined with 8.2% Nycodenz (mixed with 30% Nycodenz stock solution and granule bound synthase (GBSS)/A), a little GBSS/B was added to the solution, and it was centrifuged for 17 minutes at 1500 × g. The cells at the interface were collected and washed twice with GBSS/B (centrifuged at 500 × g for seven minutes). The final cell isolate was suspended in hepatic stellate cell medium (Kordes et al., 2014).

An immunofluorescence assay was performed to observe and identify hepatic stellate cells. Following a standard method of inoculating coverslips, the cells were fixed with 4% paraformaldehyde for 20 minutes, permeated with 0.5% Trixon X-100 for five minutes, and incubated with 5% bovine serum albumin for one hour to prevent non-specific staining. Subsequently, the primary anti-α-SMA (1:200, Abcam, Cambridge, UK) was added and incubated at 4°C for 24 hours. Alexa Fluor 488 goat anti-rabbit secondary antibody (1:1000, Abcam, Cambridge, UK) was then added for 30 minutes of incubation at 37°C. The cells were then stained with 4’,6-diamidino-2-phenylindole for three minutes, mounted with fluorescent anti-quenching agent, and photographed with a laser confocal microscope (Olympus, Tokyo, Japan). Ten positive staining cells were randomly selected and observed per sample.

### Cell Transfection

Hepatic stellate cells from rats with AH were transfected with miR-155 mimic, miR-155 inhibitor, siRNA targeting SOCS1, and their corresponding miR-155 negative control (NC) plasmids using Lipofectamine 2000. All these plasmids were purchased from Shanghai Beyotime Biotechnology Co. Ltd. (Shanghai, China) (Wu et al., 2017).

### Dual-Luciferase Reporter Gene Assay 

The biological prediction website microRNA.org was employed to analyze the target genes of miR-155, and dual-luciferase reporter gene assay was employed to verify that the candidate SOCS1 was a direct target gene of miR-155. The SOCS1-3’-untranslated region (UTR) sequence and the mutated SOCS1-3’-UTR sequence were synthesized. The two synthesized target gene fragments were cloned into the pmir GLO dual-luciferase reporter gene vector to construct the SOCS1-3’-UTR dual-luciferase reporter wild-type gene vector (pmir GLO-SOCS1) and its mutant vector (pmir GLO-mut-SOCS1). The recombinant vector was investigated by polymerase chain reaction (PCR), electrophoresis, and gene sequencing to prove that it had been successfully constructed. HEK-293T cells (Institute of Biochemistry and Cell Biology, Shanghai Institutes for Biological Sciences, Chinese Academy of Sciences, Shanghai, China) were respectively co-transfected with the two recombinant vectors and miR-155 mimic or miR-155 NC by using the transfection reagent Lipofectamine 2000 (Invitrogen, Carlsbad, CA, USA). After 48 hours of transfection, cells were lysed. The luciferase activity was detected on a Luminometer TD-20/20 detector (E5311, Promega, Madison, WI, USA) using a Dual-Luciferase^®^ Reporter Assay System kit (Promega, Madison, WI, USA) (Song et al., 2017).

### RNA Isolation and Quantitation

Total RNA from rat hepatic stellate cells was extracted according to the instructions accompanying the TRIzol reagent (Invitrogen, Carlsbad, California, USA). The primers of miR-155, SOCS1, p38, Jun N-terminal kinase (JNK), and extracellular regulated protein kinases (ERK) 1/2 primers were designed and synthesized by AuGCT biotechnology company (Beijing, China) (**Table 1**). The RNA was dissolved with ultrapure water treated with diethylpyrocarbonate. The absorbances at 260 and 280 nm were measured using an ND-1000 ultraviolet/visible spectrophotometer (NanoDrop Technologies Inc., Wilmington, USA) to determine the quality and concentration of the total RNA. The Takara reverse transcription kit was used to generate cDNA according to the kit instructions. U6 served as an internal reference for miR-155, and glyceraldehyde-3-phosphate dehydrogenase (GAPDH) served as an internal reference for gene expression. PCR was run with pre-denaturation at 95°C for 10 minutes, followed by 40 cycles of 94°C for 30 seconds, 59°C for 30 seconds, and 72°C for 30 seconds. The reliability of the PCR results was evaluated by a melting curve. The CT value was taken, △Ct = CT (target gene) - CT (internal reference), △△Ct = △Ct (experimental group) - △Ct (control group). The value was calculated by the relative quantitative method, and 2^-ΔΔCt^ indicated the relative expression of each gene (Wu et al., 2017).

**Table 1:** Primer sequences of RT-qPCR.

Target	Primer sequence
miR-155	F: 5’-TTAATGCTAATTGTGATAGGGGT-3’
	R: 5’-GCGGCTTAATGCTAATTGTGATA-3’
SOCS1	F: 5’-TCGTCCTCGTCTTCGTCCT-3’
	R: 5’-GAAGGTGCGGAAGTGAGTGT-3’
ERK1	F: 5’-GGACCGGATGTTAACCTTTA-3’
	R: 5’-TGGTTCATCTGTCGGATCAT-3’
ERK2	F: 5’-CGTACCTGGAGCAGTATTATGA-3’
	R: 5’-CCAGCTCCATGTCAAACTTG-3’
JNK	F: 5’-ACAGTGAGCAGAGCAGGCATAGTG-3’
	R: 5’-TCCTCCCCAAACAAAATAGAACCAC-3’
p38	F: 5’-TTGGTCTGTTGGATGTGTTTAC-3’
	R: 5’-TGGATTATGTCAGCCGAGT-3’
GAPDH	F: 5’-CAAGTTCAACGGCACAGTCAA-3’
	R: 5’-TGGTGAAGACGCCAGTAGACTC-3’
U6	F: 5’-CTCGCTTCGGCAGCACA-3’
	R: 5’-AACGCTTCACGAATTTGCGT-3’

SOCS1, suppressor of cytokine signaling; ERK, extracellular regulated protein kinases; JNK, Jun N-terminal kinase; GAPDH, glyceraldehyde-3-phosphate dehydrogenase.

### Western Blot Assay

The alcoholic hepatic stellate cells from rats were taken, immediately lysed on ice in pre-cooled cell lysis buffer solution (containing 1% protease inhibitor), and centrifuged at 8000 rpm for 30 min at 4°C. The supernatant was collected, and the protein concentration was measured with a bicinchoninic acid kit (Beyotime Institute of Biotechnology, Shanghai, China). Next, 50 μg protein was electrophoresed by 10% sodium dodecyl sulfate polyacrylamide gel and then electroblotted to a polyvinylidene fluoride membrane by semi-dry transfer. The membrane was fully blocked with 5% defatted milk. The membrane was combined with primary rabbit anti-mouse polyclonal antibodies (1:1000, Abcam, Cambridge, UK) to SOCS1 (ab9870), phosphorylated p38 (phospho T180 + Y182) (ab195049), ERK1/2 (ab54230), phosphorylated ERK1/2 (ab214036), JNK (ab179461), phosphorylated JNK (ab121856), or p38 (ab31828), followed by overnight culture at 4°C. Afterward, the secondary goat anti-rabbit horseradish enzyme marker (1:5000) was added for incubation for 2 hours, and the expression of the target proteins was detected using an enhanced chemiluminescence reagent electrochemiluminescence (ECL) developing solution. GAPDH served as the internal reference, and the ratio of the gray value of the target band to that of the internal reference band was the relative expression of the protein (Wu et al., 2017).

### Methyl Thiazolyl Tetrazolium (MTT) Assay

Under aseptic conditions, hepatic stellate cells in the logarithmic growth phase were adjusted to a cell density of about 80% and diluted with 0.25% trypsin to prepare a single-cell suspension. After being counted, cells (3 × 10^3^ to 6 × 10^3^ cells/well) were seeded in a 96-well plate and cultured in a saturated humidity incubator at 37°C with 5% CO_2_. After cells had adhered to the wall (overnight), 5 g/L of MTT solution was added into each well and incubated for four hours. Then 100 g/L dimethyl sulfoxide was added, and 10 minutes later, the absorbance values of each well were detected on a fully automatic microplate reader at 490 nm (Bio-Rad, Hercules, CA, USA). The cell viability curve was plotted, with the time point as the abscissa and the OD value as the ordinate (Xie et al., 2018).

### Flow Cytometry

For cell cycle detection (propidium iodide staining), after 48 hours of cell transfection, the cells were trypsinized, oscillated with medium, and centrifuged at 1200 rpm for 5 minutes to remove the supernatant. The cells were suspended with 0.5 mL PBS, aspirated with a 5-mL syringe, mixed into 5 mL of 70% (pre-cooled) ethanol, and then sealed at 4°C overnight. The fixed cells were collected the next day after centrifugation at 1200 rpm for five minutes, resuspended in 0.4 mL PBS, and gently oscillated. About 3 μL RNase-A was added until the final concentration reached about 50 μg/mL, and the cells were digested for 30 minutes at 37°C in a water bath. Then, 50-μL volumes of propidium iodide (PI) were added until the final concentration reached about 65 μg/mL, and the cells were placed on an ice bath and stained in darkness for 30 minutes. The cells were filtered through a 300-mesh (pore size 40–50 microns) nylon mesh, and the blue fluorescence cell cycle progression was recorded by a flow cytometer at an excitation wavelength of 352 nm (Becton, Dickinson and Company, NJ, USA) (Wu et al., 2017).

Cell apoptosis detection (Annexin V-FITC/PI double staining) was performed according to the instructions in the apoptosis detection kit (BestBio Science, Shanghai, China). Cells at the logarithmic growth phase were trypsinized, oscillated with medium, and centrifuged at 1200 rpm for 5 minutes to remove the supernatant. The cells were suspended in 400 μL of 1 × binding buffer at a concentration of approximately 1 × 10^6^ cells/mL. Next, 5 μL Annexin V-FITC was added into the cell suspension, gently mixed, and incubated for 15 minutes at 2–8°C in the dark. The PI (10-μL) was added, the combination was gently mixed at 2–8°C in the dark for 5 minutes, and the cells were filtered through a 300-mesh (the pore size was 40 to 50 micron) nylon mesh. Cell apoptosis was detected by a FACS Calibur flow cytometer at an excitation wavelength of 488 nm (Becton, Dickinson and Company, NJ, USA).

### Statistical Analysis

SPSS 21.0 (IBM Corp, Armonk, NY, USA) was adopted for statistical analysis. Data were expressed as mean ± standard deviation. A paired *t*-test was conducted to compare the paired data in two groups when the data distributions showed normality and equal variance. The unpaired *t*-test was conducted to compare unpaired designed data with normal distributions and equal variance. Data comparisons among multiple groups were performed by using one-way analysis of variance (ANOVA) and Tukey’s *post hoc* test for backtesting. Data comparison between groups at different time points was performed by repeated measurement ANOVA, and Bonferroni *post hoc* test was used for backtesting. The criterion for statistical significance was set at *p* < 0.05.

## Results

### The Physiological Indexes Were Changed in Rats With AH

The normal rats had good diet, mental, and activity statuses, and the body weight continued to grow without death. After acute gavage of the AH rats with white wine, they showed short-term behavioral arousal, followed by sedation for several hours, with piloerection and the body in a state of contracture. During the treatment, the rats showed reduced activity and lack of appetite. The weight gain of the model rats with AH was reduced, and some rats experienced body weight loss. **Table 2** shows that the levels of ALT, AST, MDA, and TBIL of AH model rats were appreciably higher than those of control rats, SOD and ALB levels were significantly lower (*p* < 0.05), and AST/ALT > 2 (*p* < 0.05). These results show that the AH model was successfully established.

**Table 2:** Blood lipid levels of rats.

Group	ALT (U/L)	AST (U/L)	ALB (g/L)	TBIL (μmol/L)	SOD (U/mL)	MDA (nmol/L)
Normal	61.63 ± 16.06	109.23 ± 35.92	47.55 ± 4.79	25.33 ± 6.62	126.33 ± 44.97	4.48 ± 12.79
AH	116.59 ± 21.02*	265.05 ± 39.19*	22.74 ± 5.44*	59.47 ± 10.27*	89.25 ± 21.84*	12.82 ± 2.71*

* p < 0.05 *vs*. normal hepatic stellate cells. The measurement data are expressed as mean ± standard deviation. An unpaired *t*-test was conducted to compare the unpaired designed data in two groups when data distribution was subject to normality and equal variance (n = 8). ALT, alanine aminotransferase; AST, aspartate aminotransferase; ALB, albumin; TBIL, total bilirubin; SOD, superoxide dismutase; MDA, malondialdehyde.

### Histology Confirmed the Successful Induction of the Rat AH Model

The results of HE staining (**Figures 1A, B**) revealed that the hepatocytes of normal rats were arranged radially around the central vein and that the cell morphology and the lobular structure were normal. However, the hepatocytes of AH model rats had cell swelling, intracellular mild balloon-like changes, and disordered lobular structure but had no obvious hepatocyte necrosis, inflammatory cell infiltration, or obvious fatty liver changes. These results are also consistent with successful establishment of the AH model.

**Figure 1:** Morphological observations of liver tissues of normal rats and AH rats. **(A)** The liver tissues of normal rats colored by HE staining (× 400). **(B)** The liver tissue of AH rats colored by HE staining (× 400).

### Hepatic Stellate Cells Were Successfully Isolated

Immunofluorescence staining showed that the α-SMA expression marker with bright green fluorescence in pointed shapes was evident in the vascular wall of normal rat liver tissues (**Figure 2**). However, a larger amount of green fluorescence was observed in the liver tissues of AH rats, and this was distributed in a sheet-like and fusiform manner (**Figure 2**), indicating the successful isolation of hepatic stellate cells.

**Figure 2:** Hepatic stellate cells were identified by employing immunofluorescence (× 200).

### miR-155 Had the Ability to Target SOCS1 in Rat Hepatic Stellate Cells

The biological prediction website (microRNA.org) employed to analyze the target gene of miR-155 predicted SOCS1 to be a direct target gene (**Figure 3A**). The dual-luciferase reporter gene assay (**Figure 3B**) showed that miR-155 mimic significantly inhibited the luciferase activity of the SOCS1 wild-type 3’UTR in rat hepatic stellate cells (*p* < 0.05), while miR-155 mimic had no significant effect on the luciferase activity of the mutant 3’UTR (*p* > 0.05). Collectively, we found that miR-155 could specifically bind to SOCS1-3’-UTR and downregulate SOCS1 expression after transcription.

**Figure 3:** miR-155 targets SOCS1. **(A)** The predicted binding site of miR-155 on 3’UTR of SOCS1. **(B)** The activity of luciferase of SOCS1 wild-type 3’UTR and mutant 3’UTR. *p < 0.05 *vs*. hepatic stellate cells transfected with miR-155 NC. The measurement data are expressed as mean ± standard deviation and compared by unpaired *t*-test. The cell experiment was repeated three times. SOCS1, suppressor of cytokine signaling 1; UTR, untranslated region; NC, negative cell.

### Upregulated miR-155, Downregulated SOCS1, and Activated MAPK Signaling Pathway Were Detected in the Liver Tissue of Rats With AH

The level of miR-155 and the mRNA and protein expressions of SOCS1, p38, ERK1/2, and JNK in rat liver tissues were detected by RT-qPCR and Western blot assay (**Figures 4A–C**). The level of SOCS1 was downregulated in the liver tissues of AH rats compared with normal rats (*p* < 0.05). The miR-155 expression and mRNA levels of in p38, ERK1/2, and JNK were upregulated in liver tissues of AH rats compared with normal rats (*p* < 0.05). The Western blot assay revealed that the level of SOCS1 protein decreased, and the protein level and phosphorylation of p38, ERK1/2, and JNK were elevated in AH rat liver tissues (*p* < 0.05). Taken together, miR-155 was upregulated, SOCS1 was downregulated, and the MAPK signaling pathway was activated in the AH model liver tissue.

**Figure 4:** Upregulated miR-155, downregulated SOCS1, and activated MAPK signaling pathway are observed in the liver tissue of AH rats. **(A)** mRNA expression of miR-155, SOCS1, p38, ERK1/2, and JNK in rat liver tissues. **(B, C)** Protein expression of SOCS1, p38, ERK1/2, and JNK in rat liver tissue. *p < 0.05 AH *vs*. normal hepatic stellate cells. The measurement data are expressed as mean ± standard deviation and compared by an unpaired *t*-test (n = 8). SOCS1, suppressor of cytokine signaling 1; MAPK, mitogen-activated protein kinase; AH, alcoholic hepatitis; RNA, ribonucleic acid; ERK, extracellular regulated protein kinases; JNK, Jun N-terminal kinase.

### miR-155 Activated the MAPK Signaling pathway by Suppressing SOCS1 Expression in Hepatic Stellate Cells

The results of RT-qPCR and Western blot assay (**Figures 5A–C**) showed that, compared with normal cells, the mRNA and protein levels of SOCS1 were significantly decreased, whereas miR-155 expression and protein and mRNA expression and phosphorylation of p38, ERK1/2 and JNK were significantly increased in other cells (*p* < 0.05). The mRNA and protein level of SOCS1 was significantly decreased, and the mRNA and protein expression and phosphorylation of p38, ERK1/2, and JNK were raised after transfection with miR-155 mimic or siRNA-SOCS1 (*p* < 0.05). Meanwhile, miR-155 expression was increased by transfection with miR-155 mimic (*p* < 0.05) but was unaffected by transfection with siRNA-SOCS1 (*p* > 0.05). After transfection with miR-155 inhibitor, the mRNA and protein level of SOCS1 conspicuously increased, but the level of miR-155 and the mRNA and protein expression and phosphorylation level of p38, ERK1/2, and JNK were substantially reduced (*p* < 0.05). After transfection with miR-155 inhibitor + siRNA-SOCS1, the expression of miR-155 decreased (*p* < 0.05), but the mRNA and protein expression and phosphorylation level of SOCS1, p38, ERK1/2, and JNK showed no evident changes (*p* > 0.05).

**Figure 5:** miR-155 activates the MAPK signaling pathway by suppressing SOCS1 expression in hepatic stellate cells. **(A)** The level of mRNA in related genes. **(B)** The level of protein in related genes. **(C)** Western blot protein band diagram. *p < 0.05 *vs.* hepatic stellate cells of normal rats, ^#^ *p* < 0.05 *vs*. hepatic stellate cells of rats with AH and hepatic stellate cells transfected with miR-155 NC of rats with AH. The measurement data are expressed as mean ± standard deviation. Data comparisons between groups were performed using one-way ANOVA, with Tukey’s *post-hoc* test for backtesting. Cell experiments were repeated three times. RNA, ribonucleic acid; AH, alcoholic hepatitis; NC, negative cells; ANOVA, analysis of variance.

### Downregulation of miR-155 Inhibits Hepatic Stellate Cell Proliferation by Stimulating SOCS1

The viability of hepatic stellate cells was observed by MTT assay after 24, 48, and 72 h. The results (**Figure 6**) showed no significant difference in cell viability after 24 h (*p* > 0.05), while there was a significant increase in cell viability after 48 and 72 h (*p* < 0.05) compared with normal hepatic stellate cells. The cell viability was apparently increased by miR-155 mimic or siRNA-SOCS1 treatments. However, the cell viability declined down after transfection with miR-155 inhibitor, which was negated by silencing SOCS1. In summary, downregulation of miR-155 or upregulation of SOCS1 could inhibit hepatic stellate cell proliferation.

**Figure 6:** miR-155 upregulation and SOCS1 silencing promote the cell viability of hepatic stellate cells. *p < 0.05 *vs*. normal hepatic stellate cells, ^#^ *p* < 0.05 *vs*. cells without any treatment and cells treated with miR-155 NC. The measurement data are expressed as mean ± standard deviation. Data comparison between groups at different time points was performed by repeated-measures ANOVA with post-testing Bonferroni correction. The cell experiment was repeated three times.

### Downregulation of miR-155 Impedes Cell Cycle Progression by Promoting SOCS1 Expression

The results of PI single staining (**Figures 7A, B**) showed that, compared with normal hepatic stellate cells, cell cycle changes were mainly seen in the shortening of the G0/G1 phase (reduced cell number) and prolongation of the S phase (increased cell number) (*p* < 0.05). When miR-155 mimic or siRNA-SOCS1 was applied, the G0 or G1 phase was shortened (reduced cell number) and the S phase was prolonged (increased cell number). Following miR-155 inhibitor transfection, the G0/G1 phase was prolonged (increased cell number) and the S phase was shortened (reduced cell number) (*p* < 0.05), which was abrogated by addition of siRNA-SOCS1.

**Figure 7:** miR-155 upregulation and SOCS1 silencing promote the cell cycle entry of hepatic stellate cells. **(A)** Cell cycle progression of differently transfected hepatic stellate cells. **(B)** Quantitative analysis of cell cycle rate in transfected cells. *p < 0.05 *vs.* normal hepatic stellate cells, ^#^ *p* < 0.05 *vs*. cells without any treatment and cells treated with miR-155 NC. The measurement data are expressed as mean ± standard deviation. Data comparisons between different groups were performed by using one-way ANOVA, with Tukey’s *post-hoc* test for backtesting. Cell experiments were repeated three times. ANOVA, analysis of variance.

### Downregulation of miR-155 Promotes Hepatic Stellate Cell Apoptosis by Upregulating SOCS1

The result of Annexin V/PI double staining (**Figures 8A, B**) displayed that, compared with normal hepatic stellate cells, the cell apoptosis rate in modified cells was significantly decreased (*p* < 0.05). Treatments with miR-155 mimic or siRNA-SOCS1 reduced the cell apoptosis rate dramatically (*p* < 0.05). Conversely, the cell apoptosis rate significantly increased in the presence of miR-155 inhibitor (*p* < 0.05), which was abolished by additional treatment with siRNA-SOCS1. These results show that overexpression of miR-155 or silencing of SOCS1 could inhibit the apoptosis rate of hepatic stellate cells from AH rats.

**Figure 8:** miR-155 upregulation and SOCS1 silencing repress hepatic stellate cell apoptosis. **(A, B)** Cell apoptosis abilities in cells without any treatment and cells treated with miR-155 NC. *p < 0.05 vs. normal hepatic stellate cells, ^#^ *p* < 0.05 *vs*. cells without any treatment and cells treated with miR-155 NC. The measurement data are expressed as mean ± standard deviation. Data comparisons between different groups were performed by using one-way ANOVA, with Tukey’s *post-hoc* test for backtesting. Cell experiments were repeated three times. ANOVA, analysis of variance.

## Discussion

AH is one of the most severe alcohol-related liver diseases and is characterized by necroinflammation, fibrosis, steatosis, cirrhosis, and serious compromise of liver function (Pavlov et al., 2019). Chronic and excessive alcohol consumption is an important and major cause of morbidity and mortality from AH (Chacko and Reinus, 2016). Glucocorticoid treatment in conjunction with enteral nutrition is the best treatment for patients with severe acute AH (Aday et al., 2017), and abstinence from alcohol is necessary in alcoholic liver disease (Aday et al., 2017).

The present results illustrate that the non-coding miRNA miR-155 was highly expressed in the liver tissue of rats with AH induced by gavage with wine. Extensive evidence has documented that miR-155, a known regulator of inflammation, was upregulated in serum from patients with alcoholic liver injury (Bala et al., 2012), which is in line with our present results. In addition, miR-155 can promote the production of exosomes, which could disrupt the function of autophagy to exacerbate the progression of AH (Babuta et al., 2019). A previous research study has reported a positive correlation between the activation of LPS signaling and miR-155 expression, which is indeed a critical mediator of LPS signaling in hepatic stellate cells (McDaniel et al., 2014). Moreover, miR-155 also plays an important role in the promotion of alcoholic liver injury, steatosis, and inflammation (Bala et al., 2016). Furthermore, our study revealed that downregulating miR-155 could suppress the proliferation, promote the apoptosis, and retard the cell cycle progression of hepatic stellate cells. A previous study elucidated that miR-155 downregulation reduced the proliferation, migration, and invasion but elevated the apoptosis rate of psoriasis cells (Xu et al., 2017). Another study similarly demonstrated that forced overexpression of miR-155 induced cell proliferation but repressed cell apoptosis in oral squamous cell carcinoma (Fu et al., 2017). These studies indirectly support our present findings on the effects of miR-155 on hepatic stellate cell proliferation and apoptosis.

The present results also provide evidence that SOCS1 expression is suppressed in the liver tissues of rats with AH. SOCS1, a crucial regulator for cytokine and a potential therapeutic target of liver disease, is certainly involved in the pathophysiology of liver, and its expression is closely correlated with the procession of various human liver disorders (Fujimoto and Naka, 2010). Besides, SOCS1 exerts a significant salutatory function in hepatocytes such that highly expressed SOCS1 helped to limit hepatocyte damage and macrophage inflammation (Mafanda et al., 2019). On the other hand, depletion of SOCS1 in liver tissue escalates the speed of liver regeneration and makes hepatic cells vulnerable to undergoing neoplastic transformation (Khan et al., 2019). Hence, in the treatment of alcoholic liver disease, the level of SOCS1 should be upregulated to suppress the proliferation, promote the apoptosis, and retard the cell cycle progression of hepatic stellate cells. Here, we found SOCS1 to be a target gene of miR-155. Moreover, others have shown that the expression of SOCS1 could be inhibited by miR-155 to mediate the inflammation in atherogenesis (Ye et al., 2016). Also, miR-155 is known to promote the proliferation and migration of breast cancer cells by inhibiting SOCS1 (Zhang et al., 2018). Meanwhile, another study identified that miR-155 negatively targeted SOCS1 to promote cell proliferation, migration, and invasion but to inhibit cell apoptosis in anaplastic thyroid cancer (Zhang et al., 2019). Taken together, miR-155 emerges as a potent factor for the inhibition of SOCS1, which in the present context of AH promoted hepatic stellate cell proliferation but reduced cell apoptosis.

Moreover, another critical finding of this study is that miR-155 activated the MAPK signaling pathway *via* SOCS1 to promote AH progression. It was previously reported that, through the inhibition of the phosphorylation of JNK and p38, *Gentianae macrophyllae* root extract (a constituent of traditional Chinese medicine) helped to attenuate alcoholic liver disease by constraining inflammation responses (Cui et al., 2019). Others have shown that miR-155 is involved in the mediation of inflammatory response and the MAPK signaling pathway (Zhu et al., 2012). Moreover, miR-155 suppression deactivates the expression of the MAPK signaling pathway (Yin et al., 2017). Therefore, the present findings of intercorrelation between miR-155, SOCS1, and the MAPK signaling pathway in the regulation of AH are consistent with a range of previous results in other systems.

In conclusion, miR-155 targets SOCS1 to activate the MAPK signaling pathway, which ultimately inhibits the proliferation, promotes the apoptosis, and retards the cell cycle entry of hepatic stellate cells from AH rats. The present findings may have direct application to the design of future translational research for improved diagnosis and treatment of AH patients. However, several limitations of this study must be noted. On the one hand, it would be clinically relevant to detect the expression of miR-155 and SOCS1 levels in patients with different stages of AH. On the other hand, the specific role of the MAPK signaling pathway in AH has not yet been extensively studied and should be explored through treatments with a specific inhibitor or activator of the MAPK signaling pathway.

## Data Availability Statement

The raw data supporting the conclusions of this article will be made available by the authors, without undue reservation, to any qualified researcher.

## Ethics Statement

Animal experiment protocols were approved by the Experimental Animal Ethics Committee of Linyi People’s Hospital. All animal experiments were performed in accordance with the Guide for the Care and Use of Laboratory Animals published by the US National Institutes of Health. Appropriate measures were taken to minimize the use of animals as well as their suffering.

## Author Contributions

DL and PH wrote the paper and conceived of and designed the experiments. CG and WG analyzed the data. XY and SL collected and provided the samples for this study. All authors have read and approved the final submitted manuscript.

## Conflict of Interest

The authors declare that the research was conducted in the absence of any commercial or financial relationships that could be construed as a potential conflict of interest.
